# Effect Evaluation of Bronchial Artery Embolization for Hemoptysis of Lung Cancer and Changes in Serum Tumor Markers and miR-34 Levels

**DOI:** 10.1155/2022/2471039

**Published:** 2022-08-16

**Authors:** Yan Huang, Hongxiang Liang, Zhiyong Yang, Hedai Liu, Judi Xu, Ying Huang, Qian Huang, Guoying Ni, Yufeng Ni

**Affiliations:** Department of Oncology, Xinhua Hospital Chongming Branch (Chongming Hospital Affiliated to Shanghai University of Medicine and Health Sciences), Shanghai 202150, China

## Abstract

The clinical efficacy, serum tumor markers, and miR-34 expression levels of bronchial artery embolization (BAE) in patients with lung cancer with hemoptysis are investigated. 92 patients with lung cancer hemoptysis treated in our hospital from January 2019 to December 2021 are randomly selected, and 92 patients are randomly divided into the conservative group and the BAE group according to the number table method, with 46 patients in each group. The efficacy, overall survival (OS) rate, coagulation function, hemoptysis volume, serum tumor markers, and miR-34 expression are compared among all groups at different time points. The experimental results show that the BAE treatment can promote the expression of miR-34 and inhibit the expression of tumor markers, so it can improve the efficacy of patients with lung cancer hemoptysis, improve the symptoms of hemoptysis and coagulation function, and prolong the life cycle of patients.

## 1. Introduction

Lung cancer is a common clinical malignant tumor disease, and its morbidity and mortality rank first among all kinds of malignant tumors, which pose a serious threat to the quality of life and health of patients and have become a public health problem to be solved urgently in China [1].

The pathogenesis of lung cancer is not yet clear, and it is clinically speculated to be related to factors such as environment, diet, and living habits, among which the typical clinical symptom is hemoptysis, which is characterized by rapid onset and rapid progression, leading to death or asphyxia of patients due to excessive blood loss [2]. Clinical application of current auxiliary diagnosis work includes organizing cytology and imaging examinations, but affected by technical conditions, it remains low sensitivity, low specific degree, and inspection defects such as trauma. In order to improve the clinical symptoms of lung cancer diagnosis and curative effect assessment, the diagnosis of serum tumor markers has been widely used as a reference indicator in recent years, and it will not cause obvious trauma to the body. It is a hot research direction in clinical malignant tumor treatment [3]. MicroRNAs (miRs) are small single-stranded noncoding RNA molecules, about 22 nucleotides in length, which are involved in the process of gene transcription and are related to the development of many types of cancer. Among them, miR-34 is abnormally expressed in breast cancer and prostate cancer and plays an important role. miR-34 expression is closely associated with tumor metastasis in lung cancer [4]. Bronchial artery embolization (BAE) is a minimally invasive treatment with minimal trauma and short postoperative recovery period [5].

At present, there are few literatures studies that comprehensively analyze the efficacy of BAE in the treatment of patients with lung cancer hemoptysis and its influence on miR-34 expression level and tumor markers. Therefore, this study aims to conduct a control study by randomly selecting confirmed cases of lung cancer hemoptysis to analyze the efficacy of BAE in the treatment of patients with lung cancer hemoptysis and its influence on miR-34 expression level and tumor markers. It provides new ideas for the pathological mechanism of lung cancer and the optimization of hemoptysis treatment.

The rest of this paper is organized as follows.  Section 2 discusses related work, followed by the proposed methods and evaluation criteria designed in Section 3.  Section 4 shows the experimental results.  Section 5 summarizes the full text primary coverage and future research directions.

## 2. Related Work

Common complications include hemoptysis of lung cancer; lung cancer lesions can cause blood vessel damage and pipe burst, causing hemoptysis symptoms. The principle of traditional medicines' conservative treatment is to improve the capillary permeability and lower pulmonary pressure, which can achieve effective hemostatic treatment, but the effect of hemoptysis for vascular damage cannot meet expectations and there is a high risk of recurrence. As a result, its clinical application is limited. In the conservative group, the patients are aged from 33 to 75 years, with an average of (57.31 ± 2.22) years [6].

This study shows that the BAE group has a higher total effective rate, OS, 1 year, and gets a more effective amount of hemoptysis control effect, prompt relativeness than conservative treatment; application of BAE therapy can reduce the number of hemoptysis patients to effectively control the patient's symptoms, and effectively improve the curative effect of lung cancer patients with hemoptysis and extend the life cycle. This is consistent with previous studies [7]. An analysis of the main reasons is as follows: BAE therapy can be performed through injection in the bronchial artery embolization agent blocking blood vessels, and effective control of hemoptysis, tumor embolization agent should be in a short period of time embolism peripheral arterial blood supply, ensure the tumor tissue necrosis in a short period of time, and inhibit tumor angiogenesis. This study used the gelatin sponge particles embolization agent. This study selected gelatin sponge particles as a common embolization agent , rubber sponge particles are a kind of fibrin glue material without antigenicity, nontoxic, and capable of rapid expansion. In the application of the material during the embolization of bronchial pulmonary artery, the anastomosis branch will not cause obvious effect, but can drop the spinal cord artery embolism and the risk of low bronchial ischemia necrosis. In addition, gelatin sponge particles do not cause obvious vascular stimulation, thus promoting thrombosis and achieving the therapeutic goals of mechanical embolization and hemostasis in a short time [8]. DD and FIB are both coagulation indicators that can sensitively reflect fibrinolytic activity. Abnormal increase of FIB indicates that there is fibrinolytic hyperactivity. DD is a secondary fibrinolytic metabolite, which can reflect fibrinolytic thrombi in vivo in real time. The two coagulation indexes show a trend of first increasing and then decreasing, and the change range of the BAE group was larger. BAE treatment can play a positive role in rapid hemostasis and improve the clinical efficacy by promoting thrombosis and then increase DD and FIB indexes correspondingly, and then show a decreasing trend and change to close to the normal level at the later stage. It is suggested that BAE treatment can improve the efficacy of patients with lung cancer hemoptysis, improve the symptoms of hemoptysis and coagulation indicators, and contribute to the disease control of patients [9, 10].

Carcinoembryonic antigen (CEA) is a clinically commonly used tumor sensitive marker, mainly formed in cytoplasm, transmitted by the cell membrane and secreted in extracellular and surrounding body fluids, which can be detected in serum, gastric juice, and other body fluids. With the aggravation of patients' conditions, the level of CEA will increase correspondingly [11]. Early CA125 is commonly used in clinical diagnosis of ovarian cancer, prognosis judgment, and prediction of disease recurrence with high sensitivity and positive rate, while CA125 is highly expressed in the serum of lung cancer patients [12]. The Neuron-specific enolase (NSE) is a highly expressed rate-limiting enzyme in lung cancer tissues, which is about 30 times the normal level, and the sensitivity of NSE to the diagnosis of lung cancer is over 70% [13]. The results of this study showed that the tumor markers in both groups were significantly reduced, and the inhibitory effect of BAE treatment was better. The main reason may be that BAE can relieve the symptoms of patients with lung cancer hemoptysis more effectively, thus controlling the disease of patients, and indirectly inhibiting the expression of CEA, CA125, and NSE tumor markers.

Zhang and Chen [14] showed that miR-34 was abnormally low expressed in lung cancer and was related to the physiological processes of apoptosis and proliferation of lung cancer. Similar results were obtained in this study, miR-34 expression levels in the two groups showed an increasing trend after treatment. Combined with the analysis of clinical efficacy results, it can be found that the efficacy and symptom improvement of patients with lung cancer hemoptysis have been significantly improved after treatment, which further indicates that the patient's condition has been effectively controlled, the proliferation of tumor cells has been inhibited, and the apoptosis level has been enhanced. Analysis of its mechanism may be that miR-34 can inhibit G1 cell cycle to a certain extent, *p*53 signaling pathway is involved in and plays an important role in cell growth and apoptosis, and tumor suppressor gene *p*53 has a certain regulatory effect on miR-34 gene. Moreover, *p*53 can regulate the expression level of miR-34-related downstream proteins. miR-34a reversely regulates endogenous *p*53 activity and *P*53 mRNA expression by down-regulating silent information regulator 1(SIRTl). Furthermore, the excessive activation of *p*53 is inhibited, thus enhancing the inhibitory effect of *p*53 signaling pathway on tumor cell proliferation and promoting cell apoptosis, and the maintenance of a high level of miR-34A can continuously exert the inhibitory effect of *p*53-mediated cancer through feedback activation and regulation of upstream signals [15–17].

## 3. The Proposed Methods and Evaluation Criteria

Ninety-two patients with lung cancer hemoptysis who were diagnosed and treated in our hospital from January 2019 to December 2021 were randomly selected as the study subjects, and divided into the conservative group and the BAE group according to the random number table method, with 46 cases in each group. In the conservative group, the male to female ratio is 25/21, aged from 33 to 75 years, with an average of (57.31 ± 2.22) years. The course of disease ranged from 1 to 9 years, with an average of (5.27 ± 2.19) years. The male to female ratio of the BAE group is 27/19, aged from 33 to 75 years, with an average of (57.28 ± 2.15) years. The course of disease ranged from 1 to 9 years, with an average of (5.27 ± 2.17) years. Baseline data of all subjects show no statistically significant difference and are comparable (*P* > 0.05).

### 3.1. The Proposed Methods

#### 3.1.1. Treatment Plan

The conservative group is treated by intravenous infusion of levofloxacin injection (Yangzijiang Pharmaceutical Group Co., LTD., specification: 5 ml: 0.5 g), once a day, 0.5 g each time, and intravenous infusion of hemagglutinin from white mandala snake venom (Jinzhou Aohong Pharmaceutical Co., LTD., specification: 2 units (KU)), 2 times a day, 1 KU each time.

The BAE group is given bronchial artery embolization therapy. The specific measures are as follows: gelatin sponge particles are used as embolization agent, patients are placed in supine position, 2% lidocaine is used (Zhuhai Rundu Pharmaceutical Co., LTD., Specification: 5 ml: 86.5 mg) for local anesthesia, routine disinfection, and towel spreading. A puncture is performed in the femoral artery at the place with strongest fluctuation, 1–2 cm below the inguinal ligament, and bronchial arteriography is performed. Assisted by the monitoring of the Siemens third-generation Artis zee ceiling digital angiography machine (Wuhan Ruisida Medical Technology Co., LTD.), the catheter is sent into the shadow of the left main bronchus at the level of the 4/5 vertebral body of the chest. The pig tail tube is used for thoracic aortography to determine the opening and anastomosis position of the bronchial artery. The gelatine sponge is put into the contrast solution at 550–720 *μ*m and injected into the lesion vessels. Combined with the results of arterial angiography, the degree of embolization is determined. If necessary, the bronchial artery embolization is performed on patients with large vessels and arteriovenous fistulas using spring steel coils, and the catheter is removed after the bronchial artery is completely occluded.

#### 3.1.2. Detection of Clinical Indicators

1.8 ml of fasting venous blood from the subjects in the morning is collected before treatment, 1 month and 3 months after treatment. After full mixing, the blood is left standing at room temperature for 30 min and centrifuged at 3000 r/min speed and a 7 cm radius for 10 min. Plasma and serum samples are stored separately in the new sample cup for reserve. The level of fibrinogen (FIB) in each group is measured by the CS-1300 automatic hemagglutinin analyzer (Shanghai Mojin Medical Instrument Co., LTD.). *D* Dimer (DD) and ECLIA are used to detect NEURON-specific enolase (NSE) and carcinoembryonic antigen. CEA and tumor markers of carbohydrate cancer antigen are 125 (CA125). The amount of hemoptysis before treatment, 3 days after treatment, and 7 days after treatment are completed by professionals. The three observation time points set up in this study are labeled as *T*1–*T*3.

#### 3.1.3. Determination of miR-34 mRNA Expression Level by RT-qPCR

5 ml blood samples from patients *T*1–*T*3 are taken, clearly labeled, and stored at −80°C for examination. The total RNA is extracted by the Trizol one-step method, and cDNA is obtained by the reverse transcription reaction. The PCR conditions are as follows: predenaturation at 95°C for 3 min, denaturation at 95°C for 10 s, annealing at 58°C for 30 s, extension at 72°C for 30 s, and 40 cycles. PCR products are taken for 1% agarose gel electrophoresis. A gel scanning imager is used to put the gel into the gel. U6 is used as the standardized internal reference, and the miR-34 mRNA expression is analyzed quantitatively the by ^2−△△Ct^ method compared with the Ct method.

#### 3.1.4. Follow-Up Methods

The patients are followed up until May 2022, and the survival status and survival time of the study subjects are investigated by telephone, e-mail, and door-to-door survey.

### 3.2. Evaluation Criteria

Clinical efficacy is divided into three criteria which include significant effect, effective, and ineffective [18, 19]. For patients with active bleeding stopping without recurrence, it has significant effect; for patients with reduced hemoptysis and blood loss ≥100 ml, it is effective; for patients with hemoptysis symptoms not effectively controlled or even significantly aggravated, it is ineffective. The total effective rate is the total proportion of significant effects and effective cases.

### 3.3. Statistical Methods

SPSS 26.0 statistical software is used to process the data. The measurement data are expressed as mean ± standard deviation $\left(\bar{x}\pm s\right)$ and passed the *t*-test. The counting data are expressed by percentage and passed the *x*^*2*^ test. Multiple groups of data are tested by the *F* test. The Mauchly test is used to compare the data at different time points within the group. *P* > 0.05 indicates that the covariance matrix is full of football symmetry, and *P* < 0.05 indicates that the difference is statistically significant.

## 4. Experimental Results

### 4.1. Differences in Total Clinical Efficacy

Table 1 shows the total effective rate difference. It is clearly evident from Table 1 that the total effective rate of the BAE group is higher than that of the conservative group and the difference is statistically significant (*P* < 0.05).

### 4.2. Changes in Coagulation Indexes at Different Time Points

Table 2 shows the changes in coagulation indexes at different time points.  Figure 1 shows the changes in the coagulation index at different time points. In Figure 1, *a*, *b,* and *c* represent *P* < 0.05 compared with other time points; # represents the comparison with the conservative group, *P* < 0.05. It can be observed from Table 2 and Figure 1 that the two coagulation indexes of each group show a trend of first increasing and then decreasing in *T*1–*T*3. The trend of the BAE group is more obvious, and the difference is statistically different (*P* < 0.05).

### 4.3. Changes in Hemoptysis at Different Time Points

Table 3 shows the changes in hemoptysis at different time points.  Figure 2 shows the changes in hemoptysis at different time points. In Figure 2, *a*, *b,* and *c* represent *P* < 0.05 compared with other time points; # represents the comparison with the conservative group, *P* < 0.05. Through the above experimental results, it can be observed that the hemoptysis volume in each group shows a decreasing trend. The change trend in the BAE group is more obvious, and the data are statistically different (*P* < 0.05).

### 4.4. Changes in Tumor Marker Levels at Different Time Points

Table 4 shows the changes in tumor markers at different time points.  Figure 3 shows the changes in tumor marker levels at different time points. In Figure 3, *a*, *b*, and *c* represent *P* < 0.05 compared with other time points; # represents the comparison with the conservative group, *P* < 0.05. It can be seen from Table 4 and Figure 3 that NSE, CEA, and CA125 show a decreasing trend in each group, the change range is larger in the BAE group, and the data show statistical differences (*P* < 0.05).

### 4.5. Changes in miR-34 mRNA Expression Levels at Different Time Points

Table 5 shows the changes in miR-34 mRNA expression levels at different time points.  Figure 4 shows the changes in miR-34 mRNA expression levels at different time points. In Figure 4, *a*, *b*, and *c* represent *P* < 0.05 compared with other time points; # represents the comparison with the conservative group, *P* < 0.05. It is clearly evident from Table 5 and Figure 4 that the expression levels of miR-34 mRNA show an increasing trend in each group, the change range is larger in the BAE group, and the difference shows statistical differences (*P* < 0.05).

### 4.6. Differences in Survival and Follow-Up Results

Figure 5 shows follow-up OS survival curve. It is can be seen from Figure 5 that the overall survival rate in the BAE group is higher than that in the conservative group (*P* < 0.05).

## 5. Conclusions

All the results of this study are basically consistent with those of previous studies, which indicate that there is no significant bias in the data. However, there is still a shortage of small sample sizes in this study, and further expansion of sample sizes is required to verify the conclusions. The BAE treatment can promote the expression of miR-34 and inhibit the expression of tumor markers, so it can improve the efficacy of patients, improve the symptoms of hemoptysis and coagulation function, and prolong the survival cycle of patients. BAE treatment is worthy of clinical promotion and application.

## Figures and Tables

**Figure 1:** Changes in the coagulation index at different time points. (a) Changes of DD at different time points. (b) Changes of FIB at different time points.

**Figure 2:** Changes in hemoptysis at different time points.

**Figure 3:** Changes in tumor marker levels at different time points. (a) Changes of NSE at different time points. (b) Changes of CEA at different time points. (c) Changes of CA125 at different time points.

**Figure 4:** Changes in miR-34 mRNA expression levels at different time points.

**Figure 5:** Follow-up OS survival curve.

**Table 1:** Total effective rate difference (*n* = 46, %).

Group	Excellence	Effective	Invalid	Total effective rate
BAE group	18 (39.13)	22 (47.83)	6 (13.04)	40 (86.96)
Conservative group	14 (30.43)	18 (39.13)	14 (30.43)	32 (69.57)
*x* ^*2*^				5.974
*P*				0.015

**Table 2:** Changes in coagulation indexes at different time points (*n* = 46, $\bar{x}\pm s$).

Group	Time point	DD (*μ*g/L)	FIB (g/L)
BAE group	*T*1	451.90 ± 65.91	3.37 ± 0.67
	*T*2	565.74 ± 85.98	4.24 ± 0.68
	*T*3	468.24 ± 50.02	3.48 ± 0.48
Conservative group			
	*T*1	449.30 ± 61.21	3.36 ± 0.67
	*T*2	526.28 ± 75.13	3.95 ± 0.59
	*T*3	485.81 ± 65.44	3.57 ± 0.47
*F*_time point_		412.521	442.512
*P*_time point_		<0.001	<0.001
*F*_Time point_^*∗*^_group_		531.321	524.305
*P*_Time point_^*∗*^_group_		<0.001	<0.001

**Table 3:** Changes in hemoptysis at different time points (*n* = 46, $\bar{x}\pm s$).

Group	Time point	The amount of hemoptysis (ml)
BAE group	*T*1	221.90 ± 43.91
	*T*2	105.74 ± 15.98
	*T*3	58.24 ± 6.02
Conservative group		
	*T*1	219.30 ± 41.21
	*T*2	156.28 ± 25.13
	*T*3	105.81 ± 9.44
*F*_time point_		454.522
*P*_time point_		<0.001
*F*_Time point_^*∗*^_group_		500.223
*P*_Time point_^*∗*^_group_		<0.001

**Table 4:** Changes in tumor markers at different time points (*n* = 46, $\bar{x}\pm s$).

Group	Time point	NSE (ng/ml)	CEA (ng/ml)	CA125 (U/ml)
BAE group	*T*1	45.90 ± 13.91	15.34 ± 4.51	115.14 ± 44.48
	*T*2	9.74 ± 1.98	6.74 ± 1.38	46.54 ± 13.32
	*T*3	4.24 ± 1.02	2.24 ± 0.82	12.24 ± 3.72
Conservative group				
	*T*1	45.30 ± 14.21	15.23 ± 4.49	115.09 ± 44.53
	*T*2	16.23 ± 2.13	10.13 ± 2.04	60.33 ± 10.12
	*T*3	10.51 ± 1.44	6.31 ± 1.24	32.43 ± 6.32
*F*_time point_		413.322	401.112	465.134
*P*_time point_		<0.001	<0.001	<0.001
*F*_Time point_^*∗*^_group_		544.201	535.101	567.344
*P*_Time point_^*∗*^_group_		<0.001	<0.001	<0.001

**Table 5:** Changes in miR-34 mRNA expression levels at different time points (*n* = 46, $\bar{x}\pm s$).

Group	Time point	miR-34mRNA
BAE group	*T*1	1.70 ± 0.41
	*T*2	2.24 ± 0.52
	*T*3	2.65 ± 0.62
Conservative group		
	*T*1	1.69 ± 0.39
	*T*2	1.97 ± 0.43
	*T*3	2.24 ± 0.54
*F*_time point_		409.452
*P*_time point_		<0.001
*F*_Time point_^*∗*^_group_		573.232
*P*_Time point_^*∗*^_group_		<0.001

## Data Availability

The simulation experiment data used to support the findings of this study are available from the corresponding author upon request.
